# Landscape Planning and Image Analysis Based on Multipopulation Coevolution Particle Swarm Radial Basis Function Neural Network Algorithm

This article has been retracted.

**DOI:** 10.1155/2021/2391477

**Published:** 2021-09-24

**Authors:** Yang Wang

**Affiliations:** School of Design and Art, Xijing University, Xi'an, Shaanxi 710123, China

## Abstract

Urban landscape planning and design is not only closely related to people's living environment, but also has an important impact on urban planning and development. However, there are some problems in landscape planning and design, such as excellent cases, low reuse rate of data, discrepancy between design scheme and actual situation, and serious shortage of relevant professionals. The artificial neural network can give corresponding ways to improve and solve these problems. Therefore, this paper proposes a research on garden planning and design based on multipopulation coevolution particle swarm radial basis function neural network algorithm. Based on multipopulation coevolution particle swarm radial basis function neural network algorithm, the error between the predicted evaluation value and the actual evaluation value in the simulation experiment is less than 5%, which shows good accuracy and generalization ability in performance. And in the plant configuration simulation experiment, it can effectively evaluate the urban planning and design and put forward the corresponding adjustment scheme according to the analysis results, which is more in line with the actual needs of urban planning.

## 1. Introduction

With the development of China's economy and science, improving the living environment has become an urgent requirement and an issue of increasing concern. A good living environment not only contributes to the physical and mental health of residents but also to the sustainable development of social ecology [1]. Urban garden is one of the important parts of urban construction, which has a very important impact on urban construction and urban management [2]. Urban landscape planning and design and image analysis are the general term of landscape planning and design. Landscape planning and image design puts forward the future development direction of urban landscape planning according to the needs of urban development. Landscape design is to use art and corresponding technical means to reasonably layout and arrange the architectural, natural, and human activity areas in the garden within the specified area [3, 4]. Therefore, the key of urban landscape planning image design is how to combine technology and art in a complex landscape system to reflect the artistry of the garden on the basis of meeting the requirements of landscape planning and design. However, in the actual construction, there are still many problems to be solved between technical means and art design. Urban landscape planning and design is a complex system. Whether it is plant configuration, green space planning, or scheme evaluation, it requires a lot of image calculation and data processing [5]. In addition, the reuse rate of digital garden planning and design scheme is low, partly because the document storage is not unified and partly because the garden planning and design needs to be based on the actual environment and cannot simply copy the previous excellent planning and design scheme, which requires a lot of time for continuous data sorting and research [6, 7]. Artificial neural network has good learning ability and data processing and analysis ability. It can organize the learning of archived excellent garden planning and design schemes and select the appropriate scheme according to the actual needs.

Therefore, this paper proposes a landscape planning and image analysis research based on multiswarm coevolutionary particle swarm radial basis function neural network algorithm. The first part mainly introduces the current situation and development of landscape planning and design in China. The second part is the construction of radial basis function neural network algorithm based on multipopulation coevolution particle swarm optimization algorithm, introduces radial basis function neural network algorithm and multipopulation coevolution particle swarm optimization algorithm, and constructs the corresponding model. The third part is the radial basis function neural network algorithm based on multiswarm coevolutionary particle swarm optimization and its simulation experiment in landscape planning and design, and the experimental data are collected and analyzed.

## 2. Related Work

In recent years, although modern landscape design has a lot of creative planning and design in the combination of science, engineering technology, and artistry, there are still many problems that need to be solved in the development of landscape planning and design because of various objective reasons.

  First, in the planning and design of modern gardens, it is easy to fall into the existing experience, lack of innovative spirit, and lack of corresponding innovative consciousness in environmental protection concept and artistic expression [8, 9]. Cities in different regions of China have different humanistic characteristics and local cultural heritage and show the characteristics of the city in garden planning and design on the basis of the concept of green economy in China [10]. However, the different points of urban areas are often ignored in the actual garden planning and design, and the final scheme has a very serious homogenization phenomenon.
  Second, landscape planning and design is a combination of several professions, and relevant practitioners need to learn knowledge and skills in multiple fields and apply them reasonably in landscape design [11, 12]. However, in practice, there is currently a serious shortage of personnel with relevant professional knowledge and skills in the field of landscape planning and design, which affects the efficiency and level of the final design [13]. In addition, many high-quality garden planning and design solutions cannot be further implemented in relevant actions due to construction techniques, which has a constraining effect on the development of garden planning and design [14].
  Thirdly, there is a discrepancy between the garden planning and design scheme and the actual situation. The planning and design of gardens will essentially be the planning and design of people's living environment, so different regions have different living environments and lifestyles because of the different natural conditions [15, 16]. This requires the improvement of the design based on the actual local conditions when carrying out garden design. However, in practice, many garden planning and design will not be able to fully understand the overall local reality due to incomplete and systematic data collection, which affects the final level of garden planning and design solutions [17].

In response to the problems of garden planning and design, it has been proposed to effectively evaluate garden planning and design solutions through a scientific approach. Therefore, a combination of hierarchical analysis and ecological garden evaluation system has been proposed to evaluate garden planning, which enables a systematic analysis with less data [4]. However, it cannot make corresponding suggestions for the existing problems, while its qualitative components are more and there is a gap with the actual situation. Others have proposed to construct a diversified statistical system through methods such as cluster analysis and component analysis and landscape areas and plants for planning and design evaluation [5]. Although such a method can effectively rate landscape planning and design, it does not have the corresponding predictive capability. Therefore, it has been proposed to evaluate and predict garden planning and design using the nonlinear dynamical system of BP neural networks as well as excellent information processing and learning capabilities [18]. Although the application of BP neural networks in the field of landscape planning and design has yielded good results, their models are demanding and have problems such as local optimal solutions, which have difficulty in controlling factors in practical applications and need further improvement [19].

## 3. Construction of a Radial Basis Neural Network Algorithm Model Based on Multiple Swarm Coevolutionary Particle Swarm

BP neural networks have been applied in many aspects of garden planning and design and have achieved some good results, such as the evaluation of garden plant diversity and garden lighting planning [20]. However, the traditional BP neural network has a high demand for the corresponding conditions when constructing the model, and the model results will have great accuracy defects which are difficult to control if the corresponding conditions are not met [21]. The radial basis neural network is a multilayer feedforward neural network that can achieve convergence in a short time, and it is an approximate neural network structure based on the local response characteristics of human brain neuron cells. The radial-based neural network has the best approximation performance and global optimal performance, the network structure is simple, the training method is relatively simple and easy to operate, and the computational effort is low, which can solve the problem of BP neural network accuracy defects.

### 3.1. Radial Basis Neural Network Algorithm

The structure of radial basis neural network is mainly divided into input layer, hidden layer, and output layer, and the topology of radial basis neural network is shown in Figure 1 [22]. The main role of the input layer is to transmit the signal that maps the input vector directly in the hidden space [23]. The implicit layer is a nonlinear mapping of the input through a radially symmetric and bidirectionally decaying mapping function, RBF, which contains hidden unit nodes, the number of which varies according to the specific problem. The output layer is mapped to the output of the implicit layer by means of a linear weighted summation. This shows that the radial basis neural network is not a single nonlinear neural network, but an organic unification of linear and nonlinear, although the nonlinear optimization strategy of the input layer to the hidden layer makes the learning speed of this part relatively slow, but the linear optimization strategy of the hidden layer to the output layer improves the learning speed of this part. Therefore, in a comprehensive comparison, the learning speed of radial basis neural network is higher than that of BP neural network, and it makes up for some problems of BP neural network.

The complexity of the radial basis neural network is mainly determined by the number of nodes contained in the hidden layer, and its mathematical model is represented as shown in

(1) $$\begin{array}{c} \hat{q}=\sum_{n=1}^{n_{c}}\omega_{n}g\left(\frac{{\left\|p-c_{n}\right\|}_{R^{n}}}{\sigma_{n}}\right), \end{array}$$

where the radial basis neural network input is denoted as *p* ∈ *R*^*n*^, and its output is denoted as $\hat{q}$, the output layer weight is denoted as *ω*_*n*_, the center of the radial basis is denoted as *c*_*n*_, its sensitive domain is denoted as *σ*_*n*_, the number of neurons in the hidden layer is denoted as *n*_*c*_, and the distance between the input and the center of the radial basis neural network is denoted as ‖*·*‖_*R*^*n*^_. The radial basis function is denoted as *g*(*·*), as shown in

(2) $$\begin{array}{c} R\left(x_{p}-c_{i}\right)=\exp\left(-\frac{1}{2\sigma^{2}}{\left\|x_{p}-c_{i}\right\|}^{2}\right). \end{array}$$

The variance of the basis function at this point is shown in

(3) $$\begin{array}{c} \sigma_{i}=\frac{c_{\max}}{\sqrt{2h}}, \end{array}$$

where *i*=1,2,…, *h*, *c*_max_ denotes the maximum distance from the determined center.

The connection weights between the implicit and output layers are calculated as shown in

(4) $$\begin{array}{c} \omega =\exp\left(\frac{h}{c_{\max}^{2}}{\left\|x_{p}-c_{i}\right\|}^{2}\right). \end{array}$$

Among them *p*=1,2,…, *P*;  *i*=1,2,…, *h*.

If any Boolean variable is denoted as *L*=(*a*_1_, *a*_2_,…, *a*_*n*_,…, *a*_*n*_hid__) and indicates by 0 or 1 that the node corresponding to the element *a*_*n*_ in the hidden layer does not exist or is present, respectively, the operation is shown in

(5) $$\begin{array}{c} \rho =\sum_{n=1}^{n_{\text{hid}}}a_{n}2^{-n_{\text{hid}}}, \end{array}$$

where *n*=1,…, *n*_hid_, 0 < *ρ* < 1. When any number is *ρ* taken and the number is in the interval (0, 1), there is a Boolean random vector corresponding to it. This shows that the Boolean vector *ρ* determined by any number can be used to determine the number of nodes in the hidden layer of the radial basis neural network. The expression for the output of the radial basis neural network corresponding to the sample at this time is shown in equation ({*p*_*i*_, *q*_*i*_}).

(6) $$\begin{array}{c} {\hat{q}}_{i}=\sum_{n=1}^{n_{\text{hid}}}a_{n}\times \omega_{n}\times g\left(\frac{{\left\|p_{i}-c_{n}\right\|}_{R^{n}}}{\sigma_{n}}\right). \end{array}$$

According to (1) and (2), it can be concluded that the learning training of a radial basis neural network is {*p*_*i*_, *q*_*i*_}(*i*=1,2,…, *M*) to determine the set of parameters for the training samples Θ={*c*_*n*_, *σ*_*n*_, *ω*_*n*_, *ρ*}, minimizing the function represented by

(7) $$\begin{array}{c} \min\varepsilon_{\text{RBF}}=\frac{1}{M}\sum_{i=1}^{M}\left|q_{i}-{\hat{q}}_{i}\right|. \end{array}$$

### 3.2. Basic Particle Swarm Algorithm and Multiple Swarm Coevolutionary Particle Swarm Algorithm

The particle swarm algorithm (PSO) is an evolutionary algorithm based on population intelligence, which has a simple structure that is easy to describe and implement, and the number of parameters to be adjusted and functions to be evaluated are relatively small, which can achieve fast convergence in the case of small population size. The PSO algorithm is based on the principle that an individual in the population can be treated as a particle in the n-dimensional space without the volume property, which has a certain speed of motion in the n-dimensional search space. The size of the speed is adjusted dynamically according to the particle's own motion experience and the motion experience of other individuals in the group, until the individuals in the group can move to the region with higher adaptation. Therefore, if there is a population of particles with the number of individuals in the *sn*-dimensional space, let the position vector of the first *i* individual particle in the space be denoted as *x*_*i*_={*x*_*i*1_, *x*_*i*2_,…, *x*_*in*_},  *i*=1,2,…, *s*, and then *X*_*i*_ bring the corresponding objective function into the corresponding evaluation value. The velocity of the microparticle is denoted as *v*_*i*_={*v*_*i*1_, *v*_*i*2_,…, *v*_*in*_}, the highest position of the particle is denoted as *y*_*i*_={*y*_*i*1_, *y*_*i*2_,…, *y*_*in*_}, and the highest position of all the individuals in the particle population is denoted as $\hat{y}=\left\{{\hat{y}}_{1},{\hat{y}}_{2},\ldots ,{\hat{y}}_{n}\right\}$; then, the PSO algorithm updates the velocity of the first *i* particle of each generation in *j*(1 ≤ *j* ≤ *n*) dimension as shown in

(8) $$\begin{array}{c} v_{ij}\left(t+1\right)=\omega v_{ij}\left(t\right)+c_{1}r_{1i}\left[y_{ij}\left(t\right)-x_{ij}\left(t\right)\right]+c_{2}r_{2i}\left[\omega_{j}\left(t\right)-x_{ij}\left(t\right)\right]. \end{array}$$

The velocity of the particle in *j* dimensional space is given by the velocity *i*=1,2,…, *sj*=1,2,…, *n* of the first *i* particle in the range [*v*_min_, *v*_max_]. The weight factor is denoted by *ω* and *ω* ∈ (0,1), and the acceleration constants are denoted by *c*_1_ and *c*_2_ and both are nonnegative constants. The acceleration constant is expressed as *r*_2_(*t*) ∈ (0,1) and *r*_1_(*t*) ∈ (0,1). The update equation for the corresponding individual particle positions is shown in

(9) $$\begin{array}{c} x_{i}\left(t+1\right)=x_{i}\left(t\right)+v_{i}\left(t+1\right). \end{array}$$

Then the highest position update formula for each individual particle movement through is shown in

(10) $$\begin{array}{c} y_{i}\left(t+1\right)=\left\{\begin{array}{cc} y_{i}\left(t\right), & \text{if }f\left(x_{i}\left(t+1\right)\right)\geq f\left(y_{i}\left(t\right)\right),\\ x_{i}\left(t+1\right), & \text{if }f\left(x_{i}\left(t+1\right)\right)<f\left(y_{i}\left(t\right)\right). \end{array}\right. \end{array}$$

The highest position through which all individuals in the particle population move is shown in

(11) $$\begin{array}{c} {\hat{y}}_{i}\left(t+1\right)=\arg\underset{y_{i}}{\min}f\left(y_{i}\left(t+1\right)\right),\;1\leq i\leq s. \end{array}$$

From equation (5), it can be concluded that the position of the first *i*$x_{ij}\left(t\right)=y_{ij}\left(t\right)={\hat{y}}_{i}\left(t\right)$ particle at this time is the highest position during its motion and also the highest position through which all individual particles in the particle population move. The velocity of the particle at this time is determined by the weight factor. When any particle in the swarm is close to the global best position, the speed of the particle will converge to 0. This indicates that all the particles in the swarm will eventually stop in the vicinity of the optimal solution in the basic PSO algorithm; i.e., there is no guarantee that the final convergence will reach the global optimum. To address this problem, the basic PSO algorithm needs to be further improved. Let the globally optimal particles be as shown in

(12) $$\begin{array}{c} y_{\tau }=\hat{y}. \end{array}$$

The velocity update formula as a global optimal particle is shown in

(13) $$\begin{array}{c} v_{\tau ,j}\left(t+1\right)=-x_{\tau ,j}\left(t\right)+{\hat{y}}_{i}\left(t\right)+\omega v_{\tau ,j}\left(t\right)+\beta \left(t\right)\left(1-2r_{2,j}\left(t\right)\right). \end{array}$$

The −*x*_*τ*,*j*_(*t*) position of the particle is reset from the previous *ω*_*j*_(*t*) position, and the orientation of the re-searched particle is implied in *ωv*_*τ*,*j*_(*t*) (9), and the scale factor, which controls the radius size of the random search, is indicated. According to *β*(*t*) in (9) and (10), the position update formula for the globally optimal particles in the particle population is shown in

(14) $$\begin{array}{c} x_{\tau ,j}\left(t+1\right)={\hat{y}}_{j}\left(t\right)+\omega v_{\tau ,j}\left(t\right)+\beta \left(t\right)\left(1-2r_{2,j}\left(t\right)\right). \end{array}$$

The basic framework of the particle swarm algorithm is illustrated in Figure 2.

Multiple populations evolve in concert with each other; i.e., they contain a main population and several other subpopulations, and each subpopulation evolves independently. Each subpopulation has population movement characteristics that are indistinguishable from other subpopulations, and individual particles in the subpopulation have representations that can identify the population to which they belong. According to these population characteristics, the subpopulations can be divided into populations, i.e., the individual *S*_*j*_ particles in a subpopulation are denoted as *X*_*j*_={*ρ*_*j*_, *x*_*i*1_,…, *x*_*in*_}, where the *ρ*_*j*_ is the location component of a particular population and the *x*_*in*_ the free location component. After each evolutionary iteration, the best particles of each subpopulation will be copied to the main population for the evolution of the main population, and the best particles of the main population will be obtained. After the best particle is obtained, the master population feeds the information back to the subpopulations, and each subpopulation modifies and evolves the particle movement speed based on the feedback information.  Figure 3 shows the information exchange diagram of the multipopulation coevolutionary particle swarm algorithm.

The evolutionary capacity of the population after 2 population-level evolutionary operations can be expressed by the efficiency of the best particle adaptation value enhancement in the population, as shown in

(15) $$\begin{array}{c} A\left(t\right)=\frac{f_{\max}\left(t\right)-f_{\max}\left(t-T\right)}{f_{\max}\left(t\right)}, \end{array}$$

where *f*_max_(*t*) denote the *t* adaptation value of the best particle in the population after the population has evolved for several iterations. Let the threshold of the evolutionary capacity of the population be a small positive number *ε*. If *A*(*t*) > *ε*, then the population is a growing population, and if vice versa, the population is a mature population. When the population becomes a mature population, the best individual in the population is the super individual, and the set is composed of super individuals. When the set of super individuals reaches a predefined number, the new super individuals will replace the super individuals with the smallest adaptation value in the original set of super individuals, and the set of super individuals will be reordered according to the adaptation value.

### 3.3. Radial Basis Neural Network Algorithm Model Based on Multiple Swarm Coevolutionary Particle Swarm

The framework of the algorithm based on multiple swarm coevolutionary particle swarm radial basis neural network is shown in Figure 4. The first step is to encode. If the radial basis neural network has *n*_*c*_ one hidden layer neuron, the particles are denoted as *X*_*i*_={*ρ*_*i*_, *c*_*n*_^*i*^, *σ*_*n*_^*i*^, *ω*_*n*_^*i*^} and *n*=1,2,…, *n*_hid_;  *ρ*_*i*_ ∈ (0,1). The number of nodes in the hidden layer is determined by a *ρ*_*i*_ unique Boolean variable, the *c*_*n*_^*i*^ RBF center of the neuron in the first hidden layer, *nσ*_*n*_^*i*^ width of the RBF, and the *ω*_*n*_^*i*^ connection weights between the nodes in the hidden and output layers.

The next step is to initialize the population, i.e., to determine the corresponding number of initialized populations with *M* random numbers *ρ*_*i*_ uniformly distributed in the interval (0, 1) on the basis of ensuring a uniform distribution of the population in space. In each population, three to five individual particulate initial position and velocity vectors are generated arbitrarily, whose lengths are denoted as (1+*m*+*k*)*n*_hid_, *m* and *k* output dimensions, respectively.

The third is the selection of the adaptation value, which is calculated for individual particles as shown in

(16) $$\begin{array}{c} J\left(a_{1},a_{2},\ldots ,a_{n_{\text{hid}}},c,\sigma ,\omega \right)=\ln\;\varepsilon_{\text{RBF}}+\lambda \frac{n_{\text{hid}}}{N}=\ln\;\varepsilon_{\text{RBF}}+\frac{\lambda }{N}\sum_{n=1}^{n_{\text{hid}}}a_{n}. \end{array}$$

The fourth is to perform intrapopulation particle evolution, i.e., to update individual particle movements within a population by means of multiple population coevolution particle population algorithms.

The fifth is the evolutionary iteration at the mature population level, where the algorithm ends and outputs the optimal solution when the super individual with the best adaptation value in the set of super individuals becomes the global optimal solution and the adaptation value reaches the desired requirement or the set number of iterations.

## 4. Simulation Experimental Results Based on Multiple Swarm Coevolutionary Particle Swarm Radial Basis Neural Network Algorithm in Garden Planning and Design

### 4.1. Training Results of Radial Basis Neural Network Algorithm Model Based on Multiple Swarm Coevolutionary Particle Swarm

The two-dimensional nonlinear system selected for identification in this paper is shown in

(17) $$\begin{array}{c} Y_{p}=\cos\left(2\pi k_{1}m+2\pi k_{2}n\right)\sin\left(2\pi k_{2}n\right). \end{array}$$

In 0 < *m*, *n* < 36, *k*_1_=0.04, *k*_2_=0.02, when *m* ∈ (0,36), *n* ∈ (0,36) 180 sets of data are {*q*, *m*, *m*} generated in the interval, one hundred sets of data are used as training samples and the other ninety sets of data are used as test samples. As shown in Figures 5 and 6, the training results of BP neural network algorithm, radial basis neural network algorithm, and radial basis neural network algorithm based on multiple population coevolutionary particle swarm are compared. The number of hidden layers of BP neural network algorithm, radial basis function neural network algorithm, and particle swarm radial basis function neural network algorithm based on multipopulation coevolution are 10, 10, and 6 respectively. From the results in Figure 5, it can be seen that the training time of the multipopulation coevolutionary particle swarm radial basis neural network based algorithm is longer than that of the other two algorithms, and there is no competitive advantage. However, the number of neurons in the hidden layer of the three algorithms is different, which indicates that the error of the multigroup coevolutionary particle swarm radial base neural network algorithm is reduced by an order of magnitude compared to the other two algorithms in a similar training time with a reduced number of neurons. The results in Figure 6 show that there is a significant reduction in the test error of the multigroup coevolutionary particle swarm radial basis neural network algorithm compared with the other two algorithms, which indicates that the generalization ability of the multigroup coevolutionary particle swarm radial basis neural network has improved significantly among the three algorithms.

A comparison of the fitness curves of the three algorithms for fitting a two-dimensional nonlinear function is shown in Figure 7. The yellow color indicates the BP neural network algorithm, the blue color indicates the radial basis neural network algorithm, and the purple color indicates the radial basis neural network algorithm based on multiple swarm coevolutionary particle swarm. From the curves and results, it can be seen that the convergence speed of the multipopulation coevolutionary particle swarm radial basis neural network algorithm is the fastest among the three algorithms, and it obtains better global optimal solutions than the other two algorithms.

### 4.2. Simulation Experimental Results Based on the Application of Multiple Swarm Coevolutionary Particle Swarm Radial Basis Neural Network Algorithm

Garden planning and design contains many contents, among which the planning and design of urban gardening landscape is closely related to people's life. Therefore, in the simulation experiment, this paper chooses the simulation experiment of urban garden plant landscape planning and design. In this paper, four indicators of urban landscape planning and design and image analysis are selected: sustainability of urban landscape planting, greening cost, tree species selection, and artistry of landscape planting.  Figure 8 shows the simulation results of the evaluation of urban landscape planning and design and image analysis based on multiple swarm coevolutionary particle swarm radial basis neural network algorithm in a region from 2012 to 2019. From the figure, it can be seen that the multipopulation coevolutionary particle swarm radial basis neural network algorithm can better fit the original data of urban landscape planning, and the error between the predicted and actual results is within five percent. This indicates that the prediction results and the actual results are close to the actual results based on the multigroup coevolutionary particle swarm radial basis neural network algorithm, which has strong generalization ability and can make reasonable prediction and analysis for the planning and design of the garden.

As shown in Figure 9 is the urban community garden plant landscape plan, in which 22 plant samples are arbitrarily selected in this paper, while four indicators of patch density, perimeter area ratio, spread and Shannon diversity index are selected for simulation experiments.

As shown in Figures 10 and 11, the difference curves of the four indicators of community landscaping are plotted. From the graphs, it can be seen that when the ratio of the community landscape index increases from zero, all the other three indicators except the Shannon diversity index are in a state of rapid decline, while the diversity index is increasing rapidly instead. The Shannon diversity index starts to enter a stable state when it is around 10%. But at 35%, it shows a clear downward trend again. From the results of the graph, it can be seen that the planning and design of community garden landscapes are more influenced by plant diversity, and therefore the diversity is better when the proportion is controlled between 10% and 35% in the corresponding planning and design. Of course, the content and influencing factors of garden planning and design are complicated, so it is necessary to make a value close to the upper limit of plant diversity on the basis of reasonable proportion of other influencing factors.

In summary, the multipopulation coevolutionary particle swarm radial basis neural network algorithm is able to predict and evaluate the future garden planning and design by sample training, and the error between the results and the actual results is small. Also, the simulation experiments of plant configuration show that the algorithm can effectively evaluate the existing planning scheme and give the corresponding adjustment advice based on the analysis results. However, the simulation experiments in this paper are only part of the garden planning and design, and further experiments are needed to test the performance of the multipopulation coevolutionary particle swarm radial basis neural network algorithm more comprehensively.

## 5. Conclusion

However, due to the limitations of various factors in the actual situation, there are many problems in the garden planning and design scheme, such as discrepancy with the actual situation, inconformity with the local humanistic and natural environment, and lack of professionals. At the same time, the archives of landscape planning and design are growing massively with the promotion of urban construction, but it increases the difficulty of manual management and reuse, which is not conducive to the corresponding reference of landscape planning and design. To solve the above problems, artificial neural network can provide effective ways to improve and solve them. Therefore, this paper puts forward the research of garden planning and design based on multipopulation coevolution particle swarm radial basis function neural network algorithm. Compared with other algorithms, RBF neural network algorithm based on multipopulation coevolution particle swarm optimization has low modeling requirements and can simplify the difficulty of manual operation. And it has strong data processing ability to avoid the global optimization problem of BP neural network. The application of this algorithm in landscape planning and design can solve the problems of difficult modeling, long training time, and large error with the actual evaluation value. And it can select effective data for reference according to the data in the database and provide more ideas of garden planning and design, so as to make the scheme more in line with the cultural environment of different regions. The experimental results show that when the training time of particle swarm radial basis function neural network algorithm based on multipopulation coevolution is not much different and the number of hidden layer neurons is reduced, the error result is one order of magnitude smaller than BP neural network algorithm and radial basis function neural network algorithm, and its generalization ability is greatly improved. The simulation results show that the error between the prediction results and the actual value of landscape planning and design based on multipopulation coevolution particle swarm radial basis function neural network algorithm is small and can effectively predict and analyze landscape planning and design. In addition, the algorithm can also analyze the diversity and configuration proportion of garden plants and give corresponding adjustment suggestions according to the analysis results. Landscape planning and design is a complicated project. At present, the radial basis function neural network algorithm based on multipopulation coevolution particle swarm optimization needs to be predicted and evaluated by items, and the algorithm indicators are relatively few. If the corresponding evaluation and prediction contents are added, the time and accuracy of the algorithm need to be further tested. After that, we need to continuously optimize and improve the radial basis function neural network algorithm based on multipopulation coevolution particle swarm optimization, so that it can analyze the internal relationship of data between different projects and make further analysis and evaluation.

## Figures and Tables

**Figure 1:** Topology of radial basis function neural network.

**Figure 2:** Basic framework of particle swarm optimization algorithm.

**Figure 3:** Schematic diagram of information exchange of multipopulation coevolution particle swarm optimization algorithm.

**Figure 4:** Framework diagram of particle swarm radial basis function neural network algorithm based on multipopulation coevolution.

**Figure 5:** Comparison of test error E of the three algorithms.

**Figure 6:** Comparison of test error E results of the three algorithms.

**Figure 7:** Comparison of fitness curves of three algorithms for fitting two-dimensional nonlinear functions.

**Figure 8:** Prediction results of particle swarm radial basis function neural network algorithm based on multipopulation coevolution.

**Figure 9:** Sample selection of urban garden plant landscape planning map.

**Figure 10:** Difference curve of patch density and perimeter area ratio.

**Figure 11:** Spread and diversity difference curve.

## Data Availability

The data used to support the findings of this study are available from the corresponding author upon request.
